# The Application of 5G and Artificial Intelligence Technology in the Innovation and Reform of College English Education

**DOI:** 10.1155/2022/9008270

**Published:** 2022-05-18

**Authors:** Guangya Zang, Ming Liu, Baoying Yu

**Affiliations:** ^1^School of Foreign Languages, Shijiazhuang University, Shijiazhuang 050035, China; ^2^Department of Foreign Languages, Hebei Sport University, Shijiazhuang 050041, China

## Abstract

Artificial intelligence and Fifth-Generation (5G) communication networks are examples of new information technologies that have aided and facilitated educational reform and progress. Built on the convincing requirements of college English education, with the advantage of artificial intelligence technology, we can enhance the teaching mode effectiveness, cultivate students' critical thinking ability, implement personalized wisdom and interactive learning, and thus realize artificial intelligence, and the effective use of 5G in English education is becoming a research hotspot area to be addressed. It is necessary to create a teaching aid system that uses a high-speed network and new type of technology. The specific techniques and measures for introducing 5G technology and artificial intelligence into higher education and English learning are discussed in this study. Students in higher education can benefit from the proposed technique by obtaining a better understanding of the subject and promoting their critical thinking skills. Finally, an experiment is performed to see how operative this technique is at teaching English when compared to traditional methods. The results are analyzed to determine that using this method is effective and boosts students' interest in learning as well as their hands-on abilities.

## 1. Introduction

Our civilization is presently rushing into a time period where artificial intelligence (AI) and people live and work together in an AI time period, thanks to the fast growth of AI technology in various aspects of life including, health, education, production, and learning systems. In this perspective, enhancing AI education is vital to offer students with the minimum level of AI awareness and understanding, as well as to better accommodate developing and learning in the modern system era. As most international students have been unable to attend college to take classes, distance learning for teaching majors became the primary form of teaching [1]. Online speaking classes, on the contrary, highlighted several issues throughout the epidemic, including the variety of the teaching audience, the complexity and variety of teaching platforms, and the challenges of executing classroom activities [2].

As time passes, teaching methods must be enriched on a regular basis. Communication is the aim of language, the demands of instructors and students in terms of teaching and learning can no longer match with the traditional approaches of teaching oral language [3]. Learners' motivation may be increased, and their speaking abilities can be improved by integrating artificial intelligence technology and 5G to build a new model of teaching the English language [4]. AI and 5G are two possibilities for the creation of more advanced educational communications systems. Machine learning, convolutional neural networks, and reinforcement learning are all emerging technologies with a lot of promise in terms of producing highly effective teaching and learning systems [5].

5G is gradually entering the forefront of civilization. The massive expansion of the 5G technology sector is assisting the emergence of a new smart education environment that is providing new challenges and opportunities to higher studies [6]. The 5G's ultra-high data transfer rate, significant connection, low latency, outstanding stability, and other technical features can help to optimize the learning atmosphere and improve learning skills. In the 5G epoch, the development of 5G teaching application solutions, the creation of 5G test environments, and the research and development of 5G united technologies, as well as the layout of 5G set-up facilities and the development of 5G public utility systems, must all be accelerated [7].

For 5G and AI developments, as well as higher education reform, we suggest soft computing techniques. In light of the characteristics of 5G technology, this study investigates the potential and risks of English education and teaching in the future 5G age and suggests reform and modernization from two essential parts of the educational mode and teaching materials. In addition, the precise methodologies and tactics for incorporating 5G technology and AI into higher education and English language instruction are discussed. Students in higher education will benefit from the proposed technique since it will improve their critical thinking skills and help them understand the subject better.

The remainder of the study is arranged as follows. The literature works related to this work are presented in Section 2. The framework of the proposed technique is explained in Section 3.  Section 4 compares the proposed technique's performance with that of traditional approaches. Finally, Section 5 concludes the proposed work.

## 2. Related Works

In the future of 5G, higher education will face both opportunities and challenges [6]. Traditional teaching methodologies, models, and topics for English majors' reading courses may not be sufficient to meet the development needs of the 5G age. Learners will rate course educators' educational qualities online in AI and 5G-based education systems, educators will rate peers by observing the class and looking at the summary detail of learners' and peers' summary information, and educators will ostensibly receive detailed feedback on the degree of teaching qualities [7]. Higher education is becoming increasingly popular among young people. Education and government institutions are becoming increasingly concerned about the quality of classroom instruction and students' educational levels. The focus of attention has always been on the higher-quality educational degrees of instructors and the reception levels of students. As a result, the development of an online classroom instructing quality evaluation system, as well as the enhancement of the current system, is a top priority. Many academics have looked into the impact of 5G and AI technology on education. Barate et al. [8] explored the use of augmented reality (AR) and virtual reality (VR) in higher education and the uptake of 5G technologies in educational contexts. Furthermore, after introducing numerous scenarios using AR/VR techniques, the major aspects of 5G in the enhancement of music education were evaluated. Lin et al. [9] looked into issues in classroom teaching with current communication technologies as well as novel classroom teaching scenarios employing 5G technology. AR immersion methods, remote front-projected holographic displays, panorama immersion video technologies, and 8K video camera shooting were all combined in their research to develop a three-order 11-step classroom instructing design based on 5G. The author of [10] assessed what is currently available to students and what can be done in the future with the introduction of 5G technology. The key properties of multimedia applications are examined for this aim. Ever and Rajan [11] looked at how the Internet of Things (IoT) and 5G technologies have been integrated into education and medicine, as well as the improvements in digital imaging, diagnostic decision-making, and therapeutic competence. The author of [12] discussed how the labor and educational sectors are fast transforming as a result of ongoing technological intervention and automation. Furthermore, a futures' imagining condition planning methodology was used to examine and guide education policymakers on how to best respond to the spectrum of possible futures. Chweya et al. [13] addressed the problems that develop in higher education institutions all over the world. The essay examined possible approaches for creating and implementing IoT initiatives as well as difficulties in higher education. Colaco and Lohani [14] employed 5G millimeter-wave bands with a resonance frequency of 25 GHz to build a tiny strip patch antenna for a higher-standard online educational system and other 5G uses. The researchers used a rectangular patch with a dielectric constant of 2.23 and a dielectric loss tangent of 0.0011 to test their hypothesis. The design was modeled and evaluated using the FEKO software. After simulation, it was determined that the antenna has a better return loss of −33.4 dB, a decent bandwidth of 3.56 GHz, VSWR, 2, a high gain of 10 dB, and a 99.5 percent antenna radiation efficiency. During ongoing lockdown situations around the globe, this recommended design is advantageous. This proposed design is useful during ongoing lockdown circumstances around the world. Similarly, in [15, 16], the authors related a new study for a blockchain-based educational system to the Internet of Things or keeping devices cryptographically safe on the web. Learners, professors, employers, developers, facilitators, and accreditors all benefitted from this study, which combined improved blockchain and IoT technology to create an effective online communication system [17].

Even though much work has been done to provide online teaching and education around the world, during the pandemic, online educational classes faced several challenges, including the diversity of the educating population, the complexity and diversity of teaching platforms, and the difficulty of performing classroom activities. Using the 5G methodology to create a distinctive design of higher education, more work is needed to improve learners' motivation and help them gain learning skills.

## 3. Proposed Method

This study proposed a soft computing technique for 5G on AI in innovation and reform of higher education. The schematic representation of the proposed method is shown in Figure 1.

### 3.1. Dataset

Kalboard 360, a learning management system, provided the academic dataset that was utilized in this study (LMS). Kalboard 360 is a multiagent learning management system (LMS) that is based on cutting-edge technology to make learning more effective. It is a cloud-based LMS with a unique approach. It was created to assist schools in using cutting-edge technology to help them better their learning. A platform like this allows users to access real-time teaching material from any device with an Internet connection. The data are gathered utilizing the experience API, a learner activity tracker tool (xAPI). The xAPI is a component of the training and learning architecture (TLA), which enables learners' progress and activities to be tracked, such as reading an study or viewing the training videos. The learner, activity, and items, which explain a learning experience, can all be determined using the experience API.

### 3.2. Preprocessing and Normalization

The data are unprocessed, with duplicate packets and incomplete data. It can be preprocessed to eliminate duplicates and redundant instances and missing data. Sample size reduction methods are used because the datasets for the educational system are so massive. Furthermore, because the database has so many features, feature extraction technologies are compulsory to avoid unimportant features. [16] The database is normalized during the preprocessing step. The first stage in normalizing is to compute the Z-score, which is calculated as

(1) $$\begin{array}{c} Z=\left[\frac{\left(R-\alpha \;\right)}{\omega }\right], \end{array}$$

where *α* denotes the mean of the data and *ω* indicates the standard deviation and *Z* is expressed as

(2) $$\begin{array}{c} Z=\frac{R-\bar{R}}{SD}, \end{array}$$

where *R* stands for the sample's mean and SD stands for the sample's standard deviation. The random sample looks like this:

(3) $$\begin{array}{c} \;Z_{k}=\beta_{0}+\beta_{1}R_{k}+\varepsilon_{k}, \end{array}$$

where *ε*_*k*_ denotes the errors that are dependent on *ω*^2^. Following that, the errors must not rely on each other, as provided below:

(4) $$\begin{array}{c} r_{k}∼\sqrt{W}\frac{r}{\sqrt{r^{2}+w-1}}, \end{array}$$

where *r* is a random variable.

Thereafter, the standard deviation is applied to normalize the movements of the variable. (5) is used to compute the moment scale deviation:

(5) $$\begin{array}{c} MS=\frac{\lambda^{ms}}{\emptyset^{ms}}, \end{array}$$

where *MS* denotes the moment scale:

(6) $$\begin{array}{c} \lambda^{ms}=E{\left(R-\alpha \right)}^{MS}, \end{array}$$

where *R* indicates a random variable and *E* denotes the expected value:

(7) $$\begin{array}{c} \emptyset^{ms}={\left(\sqrt{E{\left(R-\alpha \right)}^{MS}}\right)}^{2},\\ r_{w}=\frac{ms}{\bar{R}}, \end{array}$$

where *r*_*w*_ represents the coefficient of the variance.

The feature scaling procedure will be terminated by setting all of the variables to 0 or 1. The unison-based normalizing approach is the name for this procedure. The normalized equation looks like this:

(8) $$\begin{array}{c} R^{\prime }=\frac{\left(r-r_{\min}\right)}{\left(r_{\max}-r_{\min}\right)}. \end{array}$$

The data could be maintained once the data have been normalized, and the data's range and inconsistency may remain consistent. The goal of this phase is to eliminate data delay. The normalized information could then be fed into the future stages as an input.

### 3.3. Feature Extraction Using Principal Component Analysis

PCA is a statistical approach for transforming an original dataset into a new, lower-dimensional dataset. The initial dataset, which contains possibly correlated variables, is transformed into a collection of linearly uncorrelated variables. PCA is one of the most often used dimensionality reduction algorithms [18]. Initially, the data are transformed into standardized data with a mean of zero. The covariance matrix is built to generate eigenvectors and eigenvalues, which is the goal of obtaining the principal components. The primary component of new data with the highest eigenvalue is treated as the eigenvector with the highest eigenvalue, indicating the most significant link between input features. PCA is the most extensively used technique as one of the successful feature reduction methods because it is less vulnerable to diverse datasets than other holistic approaches; it is a better choice. The primary steps for turning an initial dataset *X* of *l* dimensions with possibly associated features into a new dataset based on PCA are as follows. *Z* of lower dimension *m* (*m* < *l*) is with linear uncorrelated characteristics:

(i) **Compute mean:** get the mean of each characteristic from the already processed data using
  (9) $$\begin{array}{c} \mu =\frac{1}{n}\sum_{i=1}^{n}x_{i}. \end{array}$$
(ii) **Calculate variance:** to analyze and deviation of each feature in the dataset, we use (10) to calculate variance:
  (10) $$\begin{array}{c} Var\left(X\right)=\sigma_{x}^{2},\\ =\frac{1}{n-1}\sum_{i=1}^{n}{\left(x_{i}-\mu \right)}^{2}. \end{array}$$
(iii) **Determine covariance**: (11) is used to calculate the covariance and correlation of two variables, labeled *X* and *Y*:

(11) $$\begin{array}{c} Cov\left(X,Y\right)=\sigma_{x}^{2},\\ =\frac{1}{n-1}\overset{n}{\underset{i=1}{\sum }}\left(x_{i}-\mu_{X}\right)\left(y_{i}-\mu_{Y}\right). \end{array}$$

The two features *X* and *Y* are considered independent when Cov (X, Y) = 0. PCA removes high noise from samples and uncorrelated properties from the generated dataset during the preprocessing step. PCA reduces high-dimensional data to low-dimensional data while maintaining key data properties that restrict overfitting. Furthermore, PCA improves classification performance by increasing feature equality by deleting related features.

### 3.4. Classification Using Artificial Neural Network

The artificial neural network (ANN) is a robust classification algorithm for modeling nonlinear operations, which is widely used to explain real-world systems. ANN is made up of several neurons that are intended to simulate the structure of neurons in the human brain to accomplish a task better through ‘learning, training, and ongoing improvement' [19]. The architecture of ANN is shown in Figure 2.

The input, hidden (middle), and output layers of neuron architectures make up ANNs. In the form of feature sets and activation values, the input layer collects numerical data with feature sets and activation values. Input data are sent to the hidden layer by linked neurons. The input neurons are gathered in the hidden layer to compute a weighted sum of the input neurons, which is then merged in the output layer using an activation (or transfer) function to produce results. Both neurons and connections can be given different weights during the learning process. The summed neurons will change mathematically in the output layer if the value of the activation function is increased beyond a threshold.

In the ANN process of feeding input data and terminating with output values, an epoch is the number of times the training functions are used to update the connection weights. The weights are compounded by the artificial neuron inputs, and the sum is provided to the output layer through an activation function. Linear, sigmoid, and hyperbolic tangent functions are the most commonly utilized activation functions [20]. The training is completed when the maximum epoch value and/or the validation tests are met. To evaluate the ANN's performance, the trained data are input into the test data.

### 3.5. 5G Joint Artificial Intelligence in Higher Education Innovation and Reform Application Design

The development of 5G communication technologies has had a tremendous effect on AI technology, which has remained clever to advancement at a rapid pace. Thanks to 5G technologies, which are distinguished by their omnipresent network and the Internet of thing and which have the potential to make a significant and helpful effect on AI. This influence may potentially be visible all around us, providing us with our first sight of AI systems. In the field of education, 5G and AI technologies are still widely used. Teachers can quickly hold the learning psychology and status of their students. Instructors and AI technologies working together could help teachers construct real schoolroom schemes built on data exploration. It also encourages the educational philosophy of teaching students according to their abilities. Different learning plans can be created for different students, different teaching approaches can be researched, and different instructional content can be created and disseminated based on the characteristics of different students.

### 3.6. Advanced Energy-Efficient Routing Algorithm

The proposed advanced energy-efficient routing method uses intelligent agents to execute effective communication. It also employs cluster formation and cluster head selection techniques to choose the most efficient and secure routing path. The steps of the proposed routing algorithm is shown in Algorithm 1.

## 4. Performance Analysis

To evaluate the performance of the proposed method, we classify the classes into three categories: beginner, intermediate, and advanced. For students of various levels, teachers make various teaching approaches. For instance, in the initial session, we prefer to avoid digging into far more detail and instead educate in brief, easy-to-understand terms. Students will be able to understand the fundamentals if this is done. The curricula could be adjusted to encourage the influence on learners' oral communication abilities while teaching intermediate and advanced pupils. If students are allowed they will be able to effectively understand what they may have read if they are given the time and space to learn at their speed. Oral education, as shown in Figure 3, should be centered on the students and promote the improvement of students' communication abilities.

The possibilities of the questions relevant to learning interest in the students' questionnaire were studied to better understand the change in students' interest in learning, as shown in Figure 4. The number of individuals who elected “very much in line” grew by 5.01% from 19.865 to 24.85% of the total number of pupils. The majority of individuals who selected comply “rose by 7.91% from 30.16% to 38.07% of the total population of persons, while the number of individuals who selected really not comply” fell by 1.49% from 5.34% to 3.86% of the total population of individuals. During the experimental teaching process, it shows how the student's zeal in learning grows with time as well as how their learning habits evolve.

Figure 5 illustrates the higher education proficiency classification. It can be concluded from the data in Figure that, in pair 1, the results of the pre-and post-tests of pupils' linguistic ability may be shown, with *t* = 3 : 046 and *F* = 0 : 004 0 : 05, respectively. This suggests a considerable change in learners' ability to understand language and exhibits a positive variation in learning. For the student's language learning abilities, the data come from the student's pre-test and post-test in pair 2. The outcomes of the students' language understanding ability pre-test and post-test show that, where *t* = 3 : 010 and the significance value *F* = 0 : 004 0 : 05, there is a substantial difference within the experimental class before and after the experiment, showing that the pupils' language comprehension level has changed considerably. The evidence provided for investigation as from pre-test and post-test of the students' language learning in pair 3 demonstrates that there is no notable change in the language assessment ability of the students in the experiment where *t* = 1 : 011 and the significance value *F* = 0 : 325 > 0 : 05. It shows that there are no substantial distinction and control conditions as well during the interaction.

## 5. Conclusions

With the widespread use of smartphones technology, people have to turn into an expert in understanding voice assistants with cutting-edge technologies such as real-time navigation, search engines, and application of artificial intelligence. As these technologies and products evolve with the passage of time, AI and education become more integrated. With the use of state-of-the-art technology, many offline physical courses can be adapted into virtual courses. The use of 5G has the potential to be a game changer for virtual-voiced learning; it has not only the potential to improve the teaching effectiveness of teachers but also the interest of students. As a result, this study explored the online English learning techniques in the context of 5G in the hopes of developing modern teaching approaches and insights. An investigation is conducted to evaluate the proposed system's performance in English learning to that of traditional learning. Results validate that expanding this scheme to study AI is helpful and enhances students' motivation to learn as well as their ability [17].

## Figures and Tables

**Figure 1:** Steps of the proposed method.

**Figure 2:** Architecture of ANN.

**Figure 3:** Correlation of inner elements.

**Figure 4:** Changes in students' interest in learning.

**Figure 5:** Paired sample test.

**Algorithm 1:** Energy-efficient routing.

## Data Availability

The publication contains the basic data for the results provided in the study.
